The article "Composite Dietary Antioxidant Index and Plasma Levels of Soluble Klotho: Insights from NHANES" was retracted in 2024. Reasons: signs of a paper mill; compromised peer review; unreliable results or conclusions.

# Composite Dietary Antioxidant Index and Plasma Levels of Soluble Klotho: Insights from NHANES

**DOI:** 10.1155/2023/3524611

**Published:** 2023-02-07

**Authors:** Huiqin He, Xin Chen, Da Miao, Hongxia Zhang, Yu Wang, Xingkang He, Xiaoli Chen, Ning Dai

**Affiliations:** ^1^Department of Gastroenterology, Sir Run Run Shaw Hospital, Zhejiang University Medical School, Hangzhou 310016, China; ^2^Department of Endoscopy Center, Sir Run Run Shaw Hospital, Zhejiang University Medical School, Hangzhou 310016, China

## Abstract

**Objectives:**

The association between dietary antioxidants and soluble Klotho (S-Klotho) levels remains unknown. We investigated to explore whether the composite dietary antioxidant index (CDAI) was associated with serum levels of S-Klotho in the middle-aged population.

**Methods:**

Eligible participants were identified from the National Health and Nutrition Examination Surveys (NHANES) from 2007 until 2016. The CDAI was calculated from the intake of six dietary antioxidants. The serum levels of S-Klotho were measured via enzyme-linked immunosorbent assay (ELISA). Generalized linear and nonlinear models were established to analyze the relationship between CDAI and S-Klotho levels.

**Results:**

Based on the S-Klotho quartiles, S-Klotho levels were higher in young women, Blacks, higher education, never smokers, lower waistlines, no medication use, and those with higher CDAI. Univariate analysis revealed that age, gender, race, smoking status, body mass index, waistline, and medication use were associated with serum levels of S-Klotho. When potential confounders were controlled, CDAI was significantly associated with S-Klotho levels. Subgroup analysis also revealed that this association remained significant in individuals who had the highest quartiles of CDAI, aged population (>60 years), male, and never smoker. A nonlinear relationship was observed between the CDAI and S-Klotho plasma concentrations.

**Conclusion:**

CDAI was positively correlated with plasma levels of S-Klotho after controlling for covariates. Further studies are needed to validate the current findings and explore the fundamental mechanisms.

## 1. Introduction

Oxidative stress is caused by the imbalance between oxidant generation and elimination, which contributes to multiple chronic diseases, such as cancer, aging, neurodegenerative, and cardiovascular diseases [1–3]. Overwhelming release of reactive oxygen and nitrogen species (RONS) [4] by endogenous and exogenous mechanisms can lead to deleterious effects, impaired immune defense, and signaling events [5, 6]. It is believed that accumulation of oxidative damage caused by RONS leads to impaired macromolecule synthesis (lipids, DNA, and proteins) and aging [7, 8]. For example, oxidative stress damages telomere attrition and impairs their capacity for repair, which accelerates aging and increases the risk of age-related diseases due to oxidative stress [9–11]. Conceptually, antioxidants have been postulated to protect biological systems from free radical toxicity, acting as scavengers of oxidants [12, 13]. Whether antioxidants improve adverse health consequences remains a hotly debated topic [14].

As an age-suppressor gene, Klotho is considered to originally extend life expectancy [15]. Mutations in Klotho resulted in shortened life spans in addition to multiple disorders resembling premature aging in humans [16–18]. In contrast, overexpression of Klotho in mice slowed down the aging process and increased life expectancy by 20% to 30% [17]. In humans, serum levels of Klotho were also decreased with age [19, 20]. Espuch-Oliver et al. demonstrated that soluble levels of Klotho were decreased in healthy-aged individuals duo to aging-related physiological declines [21]. They proposed that the soluble Klotho (S-Klotho) level through ELISA measurement could be considered a simple and meaningful marker of aging that can improve quality of life for the elderly [21]. Actually, the Klotho gene encoded several forms of Klotho protein, including membrane bound form and secreted form Klotho [22]. The membrane bound Klotho was primarily expressed in the renal distal convolution distal convoluted tubules of the kidney as well as in the brain [17]. The extracellular region of membrane bound Klotho could be released into the blood and urine by cleavage of *α*- and *β*-secretases [23]. The cleaved Klotho had pleiotropic properties and functioned as a humoral factor, known as the soluble Klotho (S-Klotho) [23]. Further, Klotho deficiency was related to multiple aging-related conditions, such as kidney disease, hypertension, and cancer [24]. Nakanishi et al. suggested that low-serum Klotho concentrations were associated with multiple preclinical disorders, such as overweight, abdominal obesity, hypertension, and hyperlipidemia [25]. Qiao et al. observed an inverse association between serum levels of S-Klotho and risk of pan-cancer [26]. Besides, serum levels of S-Klotho were also related to inflammatory cytokines and showed several protective effects. Martín-Núñez et al. found that reduced levels of S-Klotho were associated with the proinflammatory status, such as higher ratio of tumor necrosis factor-alpha/interleukin-10 and the C-reactive protein level [27]. Wu et al. also demonstrated that the serum levels of S-Klotho were significantly and inversely associated with four well-recognized inflammation-related biomarkers (white blood cell count, mean platelet volume, C-reactive protein, and uric acid) in the cohort [28]. Several experimental models demonstrated that upregulation of endogenous Klotho or exogenous administration of Klotho both could suppress renal fibrosis and maintain kidney function in chronic kidney disease [29]. Considering the protective effects of S-Klotho, we were curious about the association between S-Klotho levels and oxidative stress. Previously, Klotho was reported to downregulate oxidative stress [30]. However, whether antioxidants could influence S-Klotho levels has yet to be studied.

Composite dietary antioxidant index (CDAI) is a measure of individual antioxidant profile based on a combination of dietary antioxidants, including manganese, selenium, zinc, and vitamins A, C, and E [31]. The CDAI was developed to evaluate and reflect the overall impact of dietary antioxidants on health. Previous studies found that high CDAI was related to a decreased risk of various types of cancer [32–34]. To our knowledge, the relationship between CDAI and plasma levels of Klotho has not been evaluated. Whether or not dietary antioxidants influence S-Klotho levels remains largely unknown. In the current study, based on National Health and Nutrition Examination Survey (NHANES), we explored and evaluated the relationship between CDAI and S-Klotho in the middle-aged population.

## 2. Method

### 2.1. Study Population

The NHANES, which is a series of cross-sectional surveys, represents noninstitutionalized US civilian population (https://www.cdc.gov/nchs/nhanes/index.htm). The NHANES dataset includes demographic, socioeconomic, dietary, and health-related questionnaire data, which was collected through in-person interviews, physical and physiological examinations, and extensive and laboratory testing. NHANES was approved by the National Center for Health Statistical research ethics review committees and publicly available (https://wwwn.cdc.gov/nchs/nhanes/). We combined five NHANES cycles (NHANES 2007-2008, 2009-2010, 2011-2012, 2013-2014, and 2015-2016 cycle). The inclusion criteria were as follows: those who had complete data about age, gender, race, marital status, education, poverty, smoke status, energy intake, body measurement, waist circumference, use of medication, diabetes mellitus and dietary antioxidant intake, and S-Klotho level. Participants with missing or unknown data were excluded. During 2007-2008, 2009-2010, 2011-2012, and 2013-2014 study cycles, 13,760 individuals were selected to participate in the study. Individuals with missing information of composite dietary antioxidant index and serum S-Klotho level were excluded (*N* = 2,157). Besides, individuals with missing information of age, gender, race, marital status, education, poverty, smoke status, energy intake, body mass index (BMI), waist circumference, and medication use were also excluded (*N* = 1,210). Finally, 10,393 individuals with complete information were included in our analyses. All NHANES protocols were approved by the National Center for Health Statistics Research Ethics Review Board, and participants provided written informed consent. Since it used deidentified data without personally identifiable information, this study was exempted from Institutional Review Board review.

### 2.2. Calculation of CDAI

The calculation of CDAI was described previously and validated in another prospective cohort study [31]. In brief, six antioxidants (manganese, selenium, zinc, and vitamins A, C, and E) were standardized. The CDAI was based on the sum of these standardized consumptions. Each participant's food and nutrient intake in the NHANES dataset was recorded based on nonconsecutive two-day 24-hour dietary recalls, based on interviews. On the first day, the participants were interviewed at the NHANES Mobile Examination Center and then 3 to 10 days later via telephone. The Food and Nutrient Database for Dietary Studies of the United States Department of Agriculture was used to calculate the intake of antioxidants, micronutrients, and total energy [35]. Based on the questionnaire interview, we determined the intake of dietary supplements during the past month, including dosage, frequency, and duration of consumption [36].

### 2.3. Measurement of S-Klotho Levels

According to the description available on the NHANES website [19], the levels of S-Klotho of each participate were quantified using commercially available ELISA (IBL International, Japan) of frozen serum specimens. These frozen serum specimens were stored at −80°C at the Centers for Disease Control and Prevention. IBL ELISA for measurement of Klotho concentration in human samples had been extensively validated prior to the start of the study. Available serum samples of Klotho concentration were obtained from 40- to 79-year-old participants in NHANES. In summary, standard curves and relative signals of calibrator concentrations consistently met the manufacturer's criteria. The linearity of the assay was evaluated using two samples with very high and high Klotho concentrations. The intra-assay precision was obtained from two Klotho samples, and the reference ranges of Klotho concentration were evaluated in 114 healthy donors. In accordance with the manufacturer's protocol, all samples were analyzed in duplicate, and the final value was calculated based on the average of the two values. All results of analyses automatically transmitted to the laboratory Oracle Management System and evaluated by the area supervisor. Samples with greater than 10% duplicate findings were highlighted for repeated analysis. All the results were examined to ensure that they met the laboratory's routine acceptance standards before release.

### 2.4. Assessment of Covariates

To assess the influence of potential confounding factors, we selected several important covariates, including individual age (years), gender (male/female), race (White, non-Hispanic White/Black, non-Hispanic Black/Mexican, Mexican American/other, other Hispanic, other Race—including multiracial), marital status (no married/married), education level (grade or less/high school/some college/college or more), poverty (income-to-poverty ratio), smoking status (never/former/now smoker), total energy intake (Kcal/day), BMI, waist circumference, and use of medication.

### 2.5. Statistical Analysis

We gathered data from NHANES project via nhanesR. In order to illustrate the complexity of survey design, we incorporated clustering and stratification across analyses to reduce the probability of unequal selection and oversampling. For the categorical variables, the weighted chi-square test was used, and for the continuous variables, weighted linear regression model was adopted. To evaluate the relationship between CDAI and the level of S-Klotho, two models of linear regression were adopted. Model 1 was adjusted for age, gender, and race. Model 2 was adjusted for age, gender, and race, marital status, poverty, education, energy intake, BMI, waist circumference, smoke status, and medication use. The potential nonlinear association was investigated using a generalized additive model. A two-stage linear regression model was also used to determine the inflection point. All statistical analyses were performed using R packages and EmpowerStats. A *P* value < 0.05 was considered as statistically significant.

## 3. Results

The current study included 10,393 participants in the final analysis based on inclusion and exclusion criteria. The baseline features of included population were summarized in Table 1. Within the S-Klotho quartiles, significant differences were observed regarding age, gender, race, education status, smoking status, waist circumference, medication use, and CDAI. The individuals with higher levels of S-Klotho were younger, Black, had higher education, had never smoked, had a smaller waistline, no medication use, and had higher CDAI scores. There was no difference regarding marital status, poverty, BMI, and energy intake.

Further univariate analysis of associations between S-Klotho levels and various characteristics revealed that age, gender, smoke status, BMI, and waistline were inversely associated with levels of S-Klotho (Table 2). The Black and no medication use were positively associated with levels of S-Klotho (Table 2). There was a positive relationship between CDAI and serum levels of S-Klotho, although the relationship was not statistically significant (Table 2). After adjusting for age, gender, and race confounders, CDAI was significantly associated with S-Klotho levels (Table 3). In subgroup analysis, the positive association was more apparent in individuals with the highest quartiles of CDAI, all age groups, all gender groups, and never-smokers. Higher antioxidant intakes of vitamins A and C were significantly associated with higher levels of S-Klotho (Table 3). After controlling for additional confounders, such as marital status, poverty, education, energy intake, BMI, waist circumference, smoke status, and use of medication, CDAI was still significantly associated with S-Klotho levels (Table 3). In subgroup analysis, this positive association remained significant in individuals who had the highest quartiles of CDAI, older than 60 years, male gender, and who never smoked. Higher intake of vitamin A was significantly associated with higher levels of S-Klotho. With this relationship in mind, we further performed a threshold effect analysis using a nonlinear model. As Figure 1 and Table 4 shown, the serum level of S-Klotho increased by 3.38 pg/ml when the CDAI increased by one unit (CDAI > 1.5).

## 4. Discussion

In the current study, we demonstrated that overall antioxidant intakes, indicated by the CDAI, were positively and significantly associated with plasma levels of S-Klotho after adjusting for multiple covariates in the middle-aged population based on NHANES. In the aged, male, and never-smoking population, this positive association was more apparent. In the subgroup analysis of individual antioxidant components, a higher intake of vitamin A was significantly related to higher plasma levels of S-Klotho. Our results suggested that overall dietary antioxidants might influence serum levels of antiaging protein, S-Klotho.

The concentrations of RONS overwhelmingly contribute to oxidative stress, which leads to cell and tissue damage [37]. To maintain a steady state of biological redox, antioxidants may scavenge oxidants, which protects against oxidative stress. As a result, dietary antioxidants mitigate the damaging effects of oxidative stress and contribute to health [38]. CDAI represents comprehensive measurement of total antioxidant levels in the diet and is widely used in many studies. Proinflammatory cytokines, such as interleukin-1b and tumor necrosis factor-alpha, were inversely correlated with CDAI [39]. Several epidemiological studies showed that higher CDAI levels were significantly associated with reduced risk of various types of cancer. Wright et al. first showed that the combination of dietary antioxidants reduced the risk of lung cancer among male smokers [31]. Paragomi et al. showed that the overall levels of dietary antioxidants decreased the risk of pancreatic cancer [34]. Yu et al. reported an inverse relationship between CDAI and the risk of colorectal cancer, suggesting that antioxidants might reduce the incidence of colorectal cancer in the population [32]. Besides, dietary antioxidants were also reported to be associated with mortality, although not consistently. Wang et al. observed that higher intakes of antioxidants were associated with reduced mortality risk from all causes and cardiovascular disease in diabetic adults [40]. According to other studies, higher intakes of magnesium, zinc, selenium, and vitamins A, C, and E were inversely related to reduced mortality risk [41–43]. However, Genkinger et al. reported that no significant relationships existed between dietary intakes of vitamins C, E, and overall mortality [44].

However, evidence is limited to suggest any relationship between dietary antioxidants and levels of S-Klotho. Klotho was originally identified by Kuro-o et al. in 1997 as a potential an antiaging gene [15]. Mice deficient in Klotho had shortened life spans and multiple disorders resembling premature aging in humans, while mice with overexpression of Klotho could extend life span and slow down the aging process [16–18]. S-Klotho was cleaved by secretases from transmembrane Klotho and entered the circulatory system. In the circulation, S-Klotho served as the main functional form [16, 45]. Increasing evidence had suggested that Klotho could exert vasculo-protective effects and was critical for vascular health. Semba et al. showed that higher plasma levels of Klotho were independently associated with a reduced risk of cardiovascular disease in the community-based cohort [46]. Navarro-Gonzalez et al. found that lower serum Klotho concentrations were negatively associated with the presence and severity of coronary artery disease [47]. Recently, Pan et al. also showed that reduced baseline levels of circulating Klotho were associated with an increased risk of coronary artery disease in a prospective study [48]. Besides, a growing body of evidence also indicated that Klotho played a crucial anti-inflammation, antiaging, insulin resistance role, and prevention of age-related diseases. Serum levels of Klotho were reported to be associated with the proinflammatory status and well-recognized inflammatory biomarkers in the cohort [27]. The S-Klotho modulated the degree of insulin/insulin-like growth factor-1 signaling and Wnt pathway, in combating aging and tumor growth [49]. Kurosu et al. found that antiaging properties of Klotho were partly through the induction of insulin resistance. They observed that Klotho could inhibit insulin and IGF1 signaling to induce insulin resistance [16]. In addition, Klotho also suppressed cellular apoptosis and protected against hypoxia, oxidative stress, and cytotoxic drugs. Lim et al. reported that Klotho inhibited the phosphatidyl-inositol 3-kinase/serine-threonine kinase pathway, thereby enhancing manganese superoxide dismutase expression via FoxO3a in response to Tac-induced oxidative stress [30]. Consequently, Klotho interfered with insulin-like growth factor 1 signaling and increased resistance to oxidative stress. However, no study investigated whether dietary antioxidant intakes affected S-Klotho levels. The findings of the present study indicated that dietary antioxidants were positively associated with serum levels of S-Klotho after adjusting for covariates, especially for vitamin A. Previously, Azimzadeh et al. reported that vitamin D supplementation prevented the reduction in plasma Klotho in the elderly among a randomized, double-blinded, placebo-controlled clinical trial [50]. The underlying mechanism might be related to the presence of a vitamin D response element in the Klotho gene both in humans and mice [15, 51]. The expression of Klotho was upregulated by the binding of 1,25-dihydroxyvitamin D to the vitamin D receptor on the Klotho gene [15, 51]. However, whether vitamin A influenced the expression of Klotho required further investigations.

To the best of our knowledge, this is the first study to investigate the relationship between overall dietary antioxidants and plasma levels of S-Klotho in a population-based cohort, as well as its originality, a large sample size, representing of the noninstitutionalized U.S. population, and standardized methods of data collection are major strengths, which minimized any measurement bias. Our results indicated that CDAI was significantly associated with S-Klotho levels. Serum levels of S-Klotho increased more when CDAI score was greater than 1.5. Our findings provided some novel insights and clinical significances that increased dietary antioxidant intakes might positively modulate higher serum levels of S-Klotho, which could protect against age-related diseases. Nevertheless, the current study has some limitations. First, this study could not construct or confirm any causal inference due to its retrospective design. Second, despite adjusting for potential confounding, residual confounding may still exist, which might influence the relationship between CDAI and the level of S-Klotho. Third, it is unclear whether our findings based on the middle-aged population can be extended to younger population. Further studies are needed to determine if the benefit of dietary antioxidants can be extended to different populations.

In summary, our study demonstrated that CDAI was significantly associated with S-Klotho levels in middle-aged population after adjusting for multiple variables. The positive relationship was mainly observed in males, aged participants, and never smokers. Further studies are needed before the results can be generalized to other populations and establish the causal relationship between CDAI and S-Klotho levels based on investigation into the underlying mechanisms.

## Figures and Tables

**Figure 1:** Association of composite dietary antioxidant index with S-Klotho plasma levels.

**Table 1:** Characteristics of population based on S-Klotho plasma levels quartiles (*N* = 10,393).

Characteristic	S-Klotho level quartiles				*P* value
	Quartile 1	Quartile 2	Quartile 3	Quartile 4	
Age (years)	57.40	56.28	55.99	55.03	<0.01
Gender					<0.01
Female (%)	24.13	24.36	25.55	25.96	
Male (%)	25.40	28.04	25.60	20.96	
Race					<0.01
White (%)	25.09	27.01	25.76	22.14	
Mexican (%)	23.59	25.84	27.49	23.08	
Black (%)	24.50	20.59	20.87	34.03	
Other (%)	22.72	23.87	27.22	26.18	
Marital status					0.31
No married (%)	25.69	24.78	25.18	24.35	
Married (%)	24.26	26.73	25.77	23.25	
Education					0.01
Grade or less (%)	25.17	26.52	24.40	23.91	
High school (%)	27.40	25.03	26.37	21.19	
Some college (%)	25.12	26.62	26.32	21.94	
College or more (%)	22.34	26.11	24.86	26.69	
Poverty	3.26	3.32	3.36	3.33	0.58
Smoke					<0.01
Never (%)	22.36	25.44	25.94	26.26	
Former (%)	26.67	26.03	25.84	21.45	
Now (%)	28.30	28.08	24.04	19.58	
Energy intake (kcal/day)	1970.11	2013.07	2023.08	1989.21	0.23
BMI	29.73	29.50	29.51	29.28	0.30
Waist circumference (cm)	102.85	102.26	101.76	100.37	<0.01
Use of medication (%)					<0.01
Yes	25.73	26.71	24.87	22.69	
No	22.29	24.55	27.31	25.85	
CDAI	0.78	1.31	1.44	1.38	<0.01

CDAI: composite dietary antioxidant index; BMI: body mass index.

**Table 2:** Univariate analysis for S-Klotho plasma levels.

Characteristic	*β*	S-Klotho	*P* value
		95% CI	
Age	-2.48	(-3.18, -1.78)	<0.01
Gender (female)			
Male	-39.71	(-55.20, -24.22)	<0.01
Race (White)			
Mexican	15.33	(-6.61, 37.28)	0.17
Other	31.35	(8.97, 53.73)	0.01
Black	80.97	(54.32, 107.62)	<0.01
Marital status (no married)			
Yes	-10.74	(-27.29, 5.80)	0.20
Poverty	1.09	(-4.07, 6.26)	0.67
Education (grade or less)			
High school	-21.39	(-46.51, 3.72)	0.09
Some college	-2.60	(-26.37,21.16)	0.83
College or more	22.35	(-3.73, 48.42)	0.09
Smoke (no)			
Former	-39.01	(-55.08, -22.94)	<0.01
Now	-54.92	(-75.46, -34.38)	<0.01
CDAI	1.35	(-0.14, 2.85)	0.08
Energy intake	-0.0039	(-0.0120, 0.0042)	0.36
BMI	-1.27	(-2.47, -0.08)	0.04
Waist circumference	-1.22	(-1.78, -0.66)	<0.01
Use of medication (yes)			
No	26.12	(8.79, 43.45)	<0.01

CDAI: composite dietary antioxidant index; BMI: body mass index.

**Table 3:** Multivariate analysis of association between CDAI and S-Klotho plasma levels.

Characteristic	Model I	*P* value	Model II	*P* value
CDAI	2.95 (1.47, 4.42)	<0.001	2.56 (0.65, 4.47)	<0.01
Vitamin A	7.56 (3.44, 11.69)	<0.01	6.87 (2.89, 10.86)	<0.001
Vitamin C	10.33 (2.40, 18.26)	0.01	7.29 (-1.41, 15.99)	0.10
Vitamin E	2.92 (-4.12, 9.95)	0.41	1.75 (-6.59, 10.10)	0.68
Mg	3.82 (-3.10, 10.74)	0.28	5.47 (-2.80, 13.74)	0.19
Zinc	0.53 (-5.99, 7.06)	0.87	5.98 (-1.80, 13.77)	0.13
Se	-1.39 (-9.44, 6.65)	0.73	6.24 (-3.56, 16.05)	0.21
Stratified by CDAI (quartile)				
Q1	5.22 (-5.92, 16.37)	0.35	1.04 (-12.05, 14.14)	0.87
Q2	-3.40 (-23.20, 16.40)	0.73	-4.49 (-24.18, 15.20)	0.65
Q3	-3.04 (-18.83, -12.76)	0.70	-3.45 (-19.34, 12.45)	0.67
Q4	2.66 (0.05, 5.26)	0.04	2.78 (0.50, 5.07)	0.02
Stratified by age (years)				
<60	2.58 (0.66, 4.49)	<0.01	1.19 (-1.45, 3.83)	0.37
≥60	3.61 (0.81, 6.41)	0.01	5.92 (2.05, 9.79)	<0.01
Stratified by gender				
Female	2.72 (0.12, 5.32)	0.04	-0.09 (-3.65, 3.48)	0.96
Male	3.06 (1.26, 4.85)	<0.01	3.94 (1.93, 5.95)	<0.01
Stratified by smoke				
Never	3.53 (1.43, 5.63)	<0.01	3.34 (0.62, 6.06)	0.02
Former	0.39 (-2.69, 3.48)	0.80	1.10 (-2.68, 4.89)	0.56
Now	1.44 (-1.80, 4.67)	0.38	1.16 (-4.02, 6.35)	0.66

CDAI: composite dietary antioxidant index; BMI: body mass index. Model I: age, sex, and race were adjusted. Model II: age, sex, marital status, race, poverty, education, energy intake, BMI, waist circumference, smoke status, and medication use were adjusted.

**Table 4:** Threshold effect analysis of CDAI on S-Klotho by the two-piecewise linear regression.

Characteristic	Adjusted *β* (95% CI)	*P* value
Fitting by the standard linear model	2.56 (0.65, 4.47)	<0.01
Fitting by the two-piecewise linear model		
Inflection point		
CDAI < 1.5	0.46 (-1.9, 3.70)	0.78
CDAI > 1.5	3.38 (1.49, 5.27)	<0.01

Age, sex, marital status, race, poverty, education, energy intake, BMI, waist circumference, smoke status, and medication use were adjusted.

## Data Availability

The dataset was based on NHANES, which was publicly available and could be found below: https://www.cdc.gov/nchs/nhanes/.

## Abbreviations

CDAI: Component dietary antioxidant index
S-Klotho: Soluble Klotho
BMI: Body mass index
NHANES: National Health and Nutrition Examination Surveys
ELISA: Enzyme-linked immunosorbent assay
RONS: Reactive oxygen and nitrogen species.
